The article "Effect of catalpol on remyelination through experimental autoimmune encephalomyelitis acting to promote Olig1 and Olig2 expressions in mice" was retracted in 2023. Reasons: duplicated images; unreliable results or conclusions; concerns about the images.

# Effect of catalpol on remyelination through experimental autoimmune encephalomyelitis acting to promote Olig1 and Olig2 expressions in mice

**DOI:** 10.1186/s12906-017-1642-2

**Published:** 2017-05-02

**Authors:** Tao Yang, Qi Zheng, Su Wang, Ling Fang, Lei Liu, Hui Zhao, Lei Wang, Yongping Fan

**Affiliations:** 1 Department of Traditional Chinese Medicine, Beijing Tiantan Hospital, Capital Medical University, Beijing, 100050 People’s Republic of China; 2 School of Traditional Chinese Medicine, Beijing Key Lab of TCM Collateral Disease Theory Research, Capital Medical University, Beijing, 100069 People’s Republic of China; 3 Oncology Department, Guang An Men Hospital of China Academy of Chinese Medical Sciences, Beijing, 100053 People’s Republic of China

**Keywords:** Catalpol, Experimental autoimmune encephalomyelitis, Multiple sclerosis, Remyelination, Olig1, Olig2

## Abstract

**Background:**

Multiple sclerosis (MS) as an autoimmune disorder is a common disease occurring in central nervous system (CNS) and the remyelination plays a pivotal role in the alleviating neurological impairment in the MS. Catalpol, an effective component extracted from the Chinese herb *Radix Rehmanniae*, which has been proved protective in cerebral diseases.

**Methods:**

To determine the protective effects and mechanisms of Catalpol on MS, the mice with experimental autoimmune encephalomyelitis (EAE) were induced by myelin oligodendrocyte glycoprotein (MOG) _35–55_, as a model for human MS. Th17 cells were counted by flow cytometric (FCM). The expressions of nerve-glial antigen (NG) 2 and myelin basic protein (MBP) were measured by immunohistochemical staining. Olig1+ and Olig2+/BrdU+ cells were counted by immunofluorescence. Olig1 and Olig2 gene expressions were detected by real-time fluorescent quantitative reverse transcription (qRT) -PCR.

**Results:**

The results showed that Catalpol improved neurological function, reduced inflammatory cell infiltration and demyelination. It could decrease Th17 cells in the peripheral blood. It increased the protein expressions of NG2 and MBP in mice brains, up-regulated markedly protein and gene expressions of Olig1 and Olig2 in terms of timing, site and targets.

**Conclusions:**

These data demonstrated that Catalpol had a strong neuroprotective effect on EAE mice. Catalpol also plays a role in remyelination by promoting the expressions of Olig1 and Olig2 transcription factors.

## Background

Multiple sclerosis (MS) is characterized by local inflammation, demyelination, gliosis and neuronal destruction through T-cells and macrophages surrounding white matter in the central nervous system (CNS) [1, 2]. These are most responsible for disabilities as a result of neural dysfunction in teenagers [3–5]. Experimental autoimmune encephalomyelitis (EAE), has similar pathological and clinical manifestations to human MS, is a commonly used animal model of MS [6].

The study found that MS demyelination following endogenous oligodendrocyte precursor cells (OPCs) repopulate the lesion areas, and which differentiate into mature oligodendrocytes (OLs) to induce OPC-mediated remyelination [7]. OPCs expressed different signaling molecules in the process of differentiation, as high expression of nerve-glial antigen (NG) 2 in the stage of early proliferation and the expression of myelin basic protein (MBP) in the stage of OLs matured.

Following the stimulation of myelin-specific antibodies, macrophages and microglial cells attack myelin which is responsible for OLs death in MS/EAE. OLs are main macroglial cells existing in the gray and white matter in CNS. Therefore, promoting remyelination is an important strategy for the therapy of MS. MBP is expressed in OLs before the formation of myelin sheath which can be detected the myelin lesions [8]. The studies showed that OPCs is the expression of the cell surface glycoprotein NG2 [9] and the NG2 has proved to be one of the most reliable and widely-used markers for OPCs in the CNS [10–12]. Moreover, the NG2 is a kind of cells that have the capacity to generate OLs in both the developing and adult CNS [13], which is reacted to demyelination by pronounced proliferation in EAE [14]. OLs are derived from OPCs, which are a subtype of glial cells [15]. OPCs are activated by demyelination and are necessary for remyelination [16, 17]. Indeed, the scenarios of OPCs actively proliferate, migrate, differentiate and recruited to the area of damage was involved in MS. However, the capacity of it was limited. Thus, promoting the capacity of it could be a novel therapy for the treatment of MS.

MS is a major demyelinating disease of the CNS leading to functional deficits. There is no efficient treatment that can entirely prevent the disability and other clinical symptoms of MS, although the corticosteroid hormone and interferon beta are widely used in the acute and remission stage [18, 19]. Nevertheless, these therapies have potentially side-effects [20]. Traditional Chinese medicine (TCM) can be used to treat the complex and varied presentations of MS, with few side-effects [21, 22]. Catalpol belongs to iridoid, an effective component extracted from the Chinese herb *Radix Rehmanniae*. The previous studies showed the formulas were composed of *Radix Rehmanniae* such as Bu Shen Yi Sui Capsules [22–24], Liuwei Dihuang Pills [25], Zuogui pills and Yougui pills [26–28] had positive effects on neuroprotective and immune-regulation in MS/EAE. Our previous study proved Catalpol could induce OPC-mediated remyelination in vitro, which indicates that Catalpol possesses the potential ability of remyelination [29]. Consequently, the potential remyeliantion ability of Catalpol is considered as a putative target in this study in vivo. Catalpol has protective effects in cerebral diseases caused by diabetes [30, 31] and ischemia [32, 33], it has been shown to have long-term, neuroprotective properties in gerbils with transient global cerebral ischemia [32, 33]. It can inhibit apoptosis and attenuate oxidative damage to protect neurons from injury in ischemia [34–37]. It also performs neuroprotective effects by ameliorating age-related neuroplasticity loss [38]. It was recently reported that Catalpol could improve memory impairments in mice with memory loss and energy metabolism disturbance [39, 40] However, the effects and mechanisms of Catalpol in EAE have not been extensively investigated.

The experiments were conducted to investigate whether Catalpol could protect against demyelination in the acute stage and remission stage within an EAE model. The study also revealed Catalpol plays a role in remyelination by promoting the expressions of Olig1 and Olig2 transcription factors.

## Methods

### Animals

One hundred twenty female C57BL/6 mice of specific pathogen-free grade, aged 7–8 weeks and weighing 16–22 g, were provided by Beijing Vital River Laboratories, China [certification NO. SCXK (JING) 2006–0009]. The animals were kept in the Center of Laboratory Animals at Capital Medical University [certification number SYXK (JING) 2010–0020]. The experiments were approved by the Ethics Committee of Capital Medical University (No. 2011-X-001).

### Drugs and reagents

Catalpol (C_15_H_22_O_10_) was purchased from Shanghai Yuanye Bio-Technology Co. Ltd. (Shanghai, China). Prednisone acetate (PA, one kind of corticosteroids widely used in MS treatment [41, 42]) was purchased from Tianjin Pacific Ocean Pharmaceutical Product Co. Ltd. (Tianjing, China). Myelin oligodendrocyte glycoprotein peptides MOG_35–55_ (MEVGWYRSPFSRVVHLYRNGK) were synthesized by Beijing SciLight Biotechnology Co. Ltd. (Beijing, China). Complete Freund’ adjuvant (CFA) and pertussis toxin (PTX) were purchased by Sigma-Aldrich (St. Louis, MO, USA). Mouse anti-CD4 FITC ﻿and anti-IL-17A PE were purchased from BD Co. Ltd. (﻿San Diego, CA, USA). Rat anti-mouse BrdU were purchased from Beijing ZSGB-Bio Co. Ltd. (Beijing, China). Rabbit anti-mouse Olig1, rabbit anti-mouse Olig2, rabbit anti-mouse MBP, rabbit anti-mouse NG2, sheep anti-rabbit-FITC and sheep anti-rat-TRITC antibodies were purchased from Abcam (Cambridge, UK). Trizol reagent was purchased from Invitrogen (Carlsbad, CA, USA). Reverse transcription kit A3500 was purchased from Promega (Madison, Wisconsin, USA). Taq DNA polymerase, buffer and DNA molecular weight marker were purchased from TaKaRa (Madison, USA). GelRed nucleic acid gel stain was obtained from Biotium (San Francisco, USA). Agarose was purchased from Biowest Agarose Regular (Spain). PCR primers were synthesized by CWbio. Co. Ltd. (Beijing, China). Sheep anti-rabbit IgG (GK400305) and DAB (K3468) were purchased from Beijing Biosynthesis Biotechnology Co. Ltd. (Beijing, China).

### Model establishment and experimental treatment

The mice were randomly divided into six groups: normal control (NC, *n* = 20), EAE model (EAE, *n* = 20), PA - treated (*n* = 20), Catalpol – H - treated (*n* = 20), Catalpol – M - treated (*n* = 20) and Catalpol – L - treated (*n* = 20). The EAE mice were injected subcutaneously with 0.2 ml emulsion, containing 50 μg MOG_35–55_ in 100 μl of normal saline (NS) and 100 μl of CFA, followed by peritoneal injections of 500 ng of PTX on Day 0 and Day 2 post-immunization (PI). The mice in NC group were given NS instead. The PA-treated EAE mice were administered NS before symptoms appeared, and then PA (6 mg/kg) was given after the disease onset. The mice in the Catalpol – H - treated EAE group, Catalpol – M - treated EAE group, Catalpol – L - treated EAE group were given oral suspensions of 80 mg/kg, 40 mg/kg, 20 mg/kg, Catalpol respectively once a day for 40 days. BrdU was dissolved in NS at a concentration of 5 mg/ml. 4 mice from each group were given peritoneal injections of BrdU (50 mg/kg) once daily for 4 consecutive days preceding sacrifice.

### Neurological function scores in mice

After the day of immunization (Day 0), the neurological function scores of EAE mice were observed daily. Paralysis was monitored and scored using the 5 point scale [43, 44]. EAE score of 0 indicated no paralysis; 1 indicated flaccid tail; 2 denoted moderate hind-limp paralysis; 3 showed complete hind-limp paralysis; 4 indicated fore-limp paralysis; and 5 denoted death.

### Sample collection

The mice were sacrificed on Day 18 (acute stage, neurological function scores at a peak) and Day 40 (remission stage, no further progress in the signs of disease) PI. Four mice from each group were anesthetized with 10% chloral hydrate (350 mg/kg body weight, intraperitoneally). 4% paraformaldehyde was used to fix the brains for hematoxylin-eosin (H&E) staining, immunohistochemical (IHC) and immunofluorescence (IF) analysis. One or two mice from each group were perfused with 2% paraformaldehyde and 2% glutaraldehyde for observation by transmission electron microscopy (TEM). Four mice from each group were anesthetized with 10% chloral hydrate, brains of mice were quickly removed, immediately frozen in liquid nitrogen, and stored at −80 °C until analysis of mRNA with real-time fluorescent quantitative reverse transcription (qRT) - PCR analyses. The peripheral blood of four mice in each group were collected and prepared for flow cytometric (FCM) analysis.

### Determining inflammatory infiltration of the Brains of Mice by H&E staining

Prepared sections (thickness, 3 μm) were dewaxed in xylene, dehydrated with gradient alcohol for 5 min each, and stained with Harris hematoxylin for 1 min, followed by eosin for 10 min for H&E staining. The sections were dehydrated in gradient alcohol, permeabilized with xylene, mounted on neutral gum. The sections were observed with light microscopy (Nikon Eclipse 80i, Tokyo, Japan). The inflammatory cell infiltration was scored as follows [45, 46]: 0, no infiltrate; 1, scattered inflammatory cells; 2, single inflammatory cells around blood vessels; 3, inflammatory cell infiltration surrounding blood vessels; 4, inflammatory cell infiltration and perivascular cuff formation, or parenchymal necrosis.

### Observation of nerve damage in brains of mice by TEM

Cross-sections (1 mm) of the intumescentia lumbalis of the brains were embedded in Epon and sectioned on a Leica EM ultramicrotome. Thin sections (thickness, 70 nm) were viewed on a TEM (JEM-1230, Japan) using a digital camera system to obtain micrographs. Ten high-power fields (×10,000) were selected in the brains (white matter) in each group. The images were analyzed by Image-Pro Plus 6.0 (Media Cybernetics, Inc., Washington, USA) and the results were expressed as area/diameter (mean) of myelin [47–49]. To measure g-ratios, five photographs from random, non-overlapping fields were account at least 50 axons.

### IHC analysis of the brains of mice

The paraffin slices were dewaxed in xylene for 15 min and dehydrated in gradient alcohol for 5 min each. The slices were treated with 3% H_2_O_2_ for 10 min at room temperature, and then washed 3 times with PBS (pH = 7.2) for 5 min each. The slices were pre-treated using heat mediated antigen retrieval with sodium citrate buffer (pH = 6) for 20 min, and washed three times with PBS. Then, the slices were incubated with primary antibody[rabbit anti-mouse MBP (1:100), rabbit anti-mouse MAP-2 (1:200) and rabbit anti-mouse NG2 (1:100)] at 4 °C overnight. Afterwards, the slices were washed 3 times with PBS and incubated with the biotin-labeled secondary antibody (sheep anti-rabbit IgG) at 37 °C for 30 min, and then washed 3 times with PBS. Color development was accomplished with 3,3’-diaminobenzidine tetrahydrochloride (DAB). Finally, the slices were dehydrated and mounted for microscopic observation. The quantitative analysis of immunohistochemical images was carried out with a NIS-Elements BR 3.0 system. For each group, five slices were obtained, with six high-power fields randomly selected from each slice. The positive results were expressed by integral optical density (IOD).

### IF analysis of the mice brains

The slices were incubated with primary antibodies: rabbit anti-mouse Olig1 (1:200); rabbit anti-mouse Olig2 (1:100) and rat anti-mouse BrdU (1:50) at 4 °C for 2 days. Afterwards, the slices were washed 3 times with PBS and incubated with the secondary antibody (sheep anti-rabbit-FITC, sheep anti-rabbit-TRITC and sheep anti-rat-TRITC) at 37 °C for 60 min, and then washed 3 times with PBS. Finally, the slices were counter-stained by DAPI and kept at 4 °C. Quantitative analysis of the images was carried out using laser confocal scanning microscopy with five high-power fields randomly selected from each slice. The results were expressed by counted positive cells.

### qRT-PCR analysis of mRNA expression of Olig1 and Olig2 in mice brains

Total RNA was isolated from approximately 50–100 mg of brains tissue using Trizol, according to the manufacturer’s instructions. The concentration of each RNA sample was measured spectrophotometrically. The integrity of RNA samples was assessed by agarose gel electrophoresis. The cDNA was synthesized from total RNA by the reverse transcription of 1 μg of total RNA. The PCR primers were designed by the Primer Premier 5.0 software, based on the Gene Bank Accession as follows: Olig1 F, **5′-**CTCTTCCACCGCATCCCTTCTCCC-**3′,** Olig1 R, **5′-**CGCTCGCGGCTGTTGATCTTGC-**3′,** Olig2 F, **5′-**TCCACCAAGAAAGACAAGAAGCAGA-**3′,** Olig2 R, **5′-**ATGGCGATGTTGAGGTCGTGC-**3′,** Mouse β-actin F, **5′-**GCCTTCCTTCTTGGGTAT-**3′** and Mouse β-actin R, **5′-**GGCATAGAGGTCTTTACGG-**3′** The amplified fragments were 162, 107 and 97 base pairs (bp), respectively. The sample reaction system (12 μl) comprised 2 μg RNA and oligo DT 1 μl, along with DEPC water. Real time reaction mixture (20 μl) contained: 10 μl of UltraSYBR Mixture (2×), 0.4 μl of the upstream primer (10 μmol/L), 0.4 μl of downstream primer (10 μmol/L), 2 μl of cDNA, and DEPC water. The relative quantification (RQ) was analyzed by the 2^-ΔΔCt^ method.

### Western blot analysis

Protein extraction (RIPA) according to the procedures specified by the manufacturers. Membranes were incubated with primarily anti-Olig1 antibody (1:2,000), anti-Olig2 antibody (1:2,000), and rabbit polyclonal anti-β-tubulin antibody (1:5,000) in blocking solution at 4 °C overnight. Data were represented by IOD ratio (ImageQuant TL 2005 image analysis software, Amersham, Biosciences, Piscataway, NJ).

### Intracellular cytokine analysis by FCM

One milliliter of venous blood was collected from each subjects into ethylenediaminetetraacetic acid (EDTA) tubes. For Th17 assay, cells were stimulated with phorbol myristate acetate (PMA 100 ng/ml) and ionomycin (1 μg/ml) with the presence of monensin (0.7 μg/ml) (BD Bioscience, USA) at 37 °C for 4 h. Blood cells were incubated with mouse anti-CD4 FITC for 30 min at 37 °C, washed with FACS buffer, fixation/permeabilization buffer for 30 min at 4 °C, and then mouse anti-IL-17A PE for 3 h at 37 °C. A control group treated with isotype control antibody was prepared. Cells were fixed in formaldehyde and then analyzed on a BD-FACS Calibur (USA). Data were analyzed based on the percentage of Th17 cells by FlowJo 7.6.1.

### Statistical analysis

The data were expressed as mean ± standard error (SE) and analyzed with SPSS version 17.0 (SPSS Inc., Chicago, IL, USA). All the data were firstly subjected to descriptive statistics for normality. The data with normally distributed and equal variances were examined using one-way ANOVA with a post-hoc LSD test, otherwise, the data were performed with a rank-sum test. The family-wise error rate was controlled by the statistical method of Bonferroni. A value of *P* < 0.05 was considered to indicate statistical significance.

## Results

### Incidence, mortality and latency of EAE in the mice

The incidence of mice with EAE was 100%. The mortality of EAE mice and Catalpol – H - treated EAE mice was 10%. The latency of Catalpol – M - treated EAE mice and Catalpol – L - treated EAE mice were significantly shorter than that of the EAE mice (*P* < 0.05, Table 1).

**Table 1:** The incidence rate, mortality rate and latency of EAE mice $\left(\overline{x}\pm \mathrm{s}\right)$

Group	Number (n)	Incidence (%)	Mortality (%)	Latency (days)
NC	20	-	-	-
EAE	20	100	10	9.50 ± 0.93
EAE + PA	20	100	0	9.86 ± 2.34
EAE + Catalpol – H	20	100	10	11.05 ± 2.71
EAE + Catalpol – M	20	100	0	12.05 ± 3.36^#^
EAE + Catalpol – L	20	100	0	12.25 ± 2.95^#^

Note: ^#^ *P* < 0.05 vs. EAE group

### Neurological function scores of the mice

Neurological impairment was visually apparent from Day 8 and all mice developed neurological deficiencies. Observed symptoms in the mice included flaccid tail, staggering, hind-limp paralysis, four-limb paralysis and even death. The average neurological function score of the EAE mice was 2.4 and reached the peak on Day 15 and Day 16. The scores declined slightly until Day 40 after the peak. The scores were decreased significantly from Day 33 to Day 39 PI in PA-treated mice, compared to EAE mice (*P* < 0.05, *P* < 0.01). The scores were decreased significantly from Day 9 to Day 17 PI, from Day 28 to Day 37 PI in Catalpol – M - treated mice, compared to EAE mice (*P* < 0.05, *P* < 0.01). The scores were decreased significantly on Day 15 to Day 16 PI in Catalpol – M - treated mice, compared to PA - treated mice EAE mice (*P* < 0.05, *P* < 0.01). The scores were decreased significantly on Day 10 and Day 13 PI in Catalpol – M - treated mice, compared to Catalpol – H, L - treated mice EAE mice (*P* < 0.05, Fig. 1)

**Fig. 1:** The neurological function scores of the mice. Results are expressed as means ± SE. The PA was given after the disease onset. The mice in the Catalpol treated groups were given oral suspensions of 80 mg/kg, 40 mg/kg, 20 mg/kg respectively once a day for 40 days. The scores were measured in NC (×), EAE (●), EAE+ PA (6 mg/kg, ◆), EAE + Catalpol–H (80 mg/kg, ▲), EAE + Catalpol–M (40 mg/kg,△) and EAE + Catalpol–L (20 mg/kg, ■). Note: ^#^ *P* < 0.05, ^##^ *P* < 0.01 vs. EAE; ^◆^ *P* < 0.05, ^◆◆^ *P* < 0.01 vs. EAE+ PA; ^△^ *P* < 0.05 vs. EAE + Catalpol– M

### Inflammatory cells infiltration in brains and spinal cord of mice

The inflammatory cells in the brains and spinal cord of mice were observed with light microscopy with H&E staining on Day 18 and 40 PI. There was a very small amount inflammatory cell in the NC group. A large number of inflammatory cells were aggregated around small blood vessels to form “sleeve-like” structures in the EAE group. Conversely, treatment with PA or high, middle and low concentrations Catalpol reduced inflammatory cell infiltration (Figs. 2 and 3). The histopathology scores significantly increased in EAE mice on Day 18 and 40 PI, compared with the NC mice (*P* < 0.01). Conversely, the treatment with PA and Catalpol reduced obviously inflammatory cell infiltration (*P* < 0.01).

**Fig. 2:** Observation of pathological changes in the brains of mice under the light microscope with H&E staining. A1 to F1 and A2 to F2 show the pathological changes in the brains of mice on Day 18 and Day 40 in NC (*n* = 4), EAE (*n* = 4), EAE+ PA (*n* = 4), EAE + Catalpol–H (*n* = 4), M (*n* = 4) and L (*n* = 4) mice, respectively (scale bar 20 μm). Note: ^**^ *P* < 0.01 vs. NC; ^##^ *P* < 0.01 vs. EAE

**Fig. 3:** Observation of pathological changes in the spinal cord of mice under the light microscope with H&E staining. A1 to D1 and A2 to D2 show the pathological changes in the spinal cord of mice on Day 18 and Day 40 in NC (*n* = 4), EAE (*n* = 4), EAE+ PA (*n* = 4), EAE + Catalpol – M (*n* = 4) mice, respectively (scale bar 20 μm)

### Nerve damage in brains of mice

Further study was carried out using TEM on Day 40 PI. The ultrastructure of myelin and axons in the brains was normal in the NC mice. However, the EAE mice showed a fluffy layer structure, axonal edema and disintegration. Demyelination was lighter in PA-treated EAE mice. Some small caliber axons were surrounded by thin myelinated sheaths in Catalpol-treated EAE mice. The damage was quantified with the ratio of area/diameter (mean) of myelin. The results showed that the ratios of in the brains of EAE mice were markedly increased compared to those of NC mice on Day 18 and 40 PI (*P* < 0.01). The treatment with PA or Catalpol at middle dosage reduced significantly the ratios on Day 18 and 40 PI (*P* < 0.05, *P* < 0.01). Catalpol at high or low dosage reduced significantly the ratios on Day 18 or 40, respectively (*P* < 0.05, *P* < 0.01, Fig. 4). PA and Catalpol at middle dosage treatments result in remyelination, as evidenced by newly formed and relatively thinner myelin sheaths (a characteristic associated with remyelination).

**Fig. 4:** Observation of pathological changes (Area/Diameter) and remyelination (g-ratio) in the brains of mice under the TEM. **a** to **f** show the demyelination in the brains of mice on Day 40 in NC (*n* = 4), EAE (*n* = 4), EAE+ PA (*n* = 4), EAE + Catalpol–H (*n* = 4), M (*n* = 4) and L (*n* = 4) mice, respectively (scale bar 1 μm). The EAE mice showed a fluffy layer structure, axonal edema and disintegration (arrows). Demyelination was lighter in PA and Catalpol-treated EAE mice (*arrows*). Note: ^*^ *P* < 0.05, ^**^ *P* < 0.01, ^***^ *P* < 0.001 vs. NC; ^#^ *P* < 0.05, ^##^ *P* < 0.01, ^###^ *P* < 0.001 vs. EAE

### FCM analysis of blood CD4 + IL-17A+ T cells

To assess the changed of pathogenic Th17 cells in EAE mice, the levels of CD4 + IL-17A + T cells were measured by flow cytometric (FCM). There was a significant increase in CD4 + IL-17A + T cells in EAE group comparing with EAE + PA group and EAE + Catalpol - M group on Day 18 and Day 40 respectively (P < 0.05) (Fig. 5).

**Fig. 5:** Effect of Catalpol on the expression of CD4 + IL-17A + T cells in the peripheral blood on Day 18 and 40 in NC (*n* = 4), EAE (*n* = 4), EAE+ PA (*n* = 4), EAE + Catalpol – M (*n* = 4) mice. Note: ^*^ *P* < 0.05 vs. NC; ^#^ *P* < 0.05, vs. EAE

### Protein expression of NG2 in the brains of mice on Day 18 and Day 40 PI

NG2 protein expressions in the brains of EAE mice were decreased on Day 18 PI compared to NC mice (*P* < 0.05). In contrast, NG2 was increased significantly in Catalpol – H, M and L - treated EAE mice compared to EAE mice in the brains on Day 18 and Day 40 (*P* < 0.01). The data also showed that NG2 in the brains of mice was increased significantly in Catalpol – H, M and L - treated EAE mice compared with the PA - treated EAE mice on Day 40 (*P* < 0.01, Fig. 6).

**Fig. 6:** The protein expressions of NG2 in the brains of mice on Day 18 and Day 40. **a** to **f** show NG2 expressions in the cortex of mice on Day 40 in NC (*n* = 4), EAE (*n* = 4), EAE+ PA (*n* = 4), EAE + Catalpol–H (*n* = 4), M (*n* = 4) and L (*n* = 4) mice, respectively (scale bar 20 μm). The protein expressions of NG2 in the cortex of mice were analyzed. Note: ^*^ *P* < 0.05 vs. NC; ^##^ *P* < 0.01 vs. EAE; ^◆^ *P* < 0.05 vs. EAE + PA; ^▲^ *P* < 0.05, ^▲▲^ *P* < 0.01 vs. EAE + Catalpol–H

### Protein expression of MBP in the brains of mice on Day 18 and Day 40 PI

The protein expression of MBP in the brains of mice was observed using IHC. On Day 18, the data showed that MBP in the cortex, lateral ventricle (LV) and hippocampal DG region of mice was significantly decreased in EAE mice compared with NC mice, respectively (*P* < 0.01). MBP increased significantly in PA, Catalpol – M and L - treated EAE mice compared with the EAE mice in the lateral ventricle (*P* < 0.05, *P* < 0.01), it increased significantly in PA - treated EAE mice compared with the EAE mice in the cortex (*P* < 0.05) and it also increased significantly in Catalpol – L - treated EAE mice compared with the EAE mice in the hippocampal DG region (*P* < 0.05). The data also showed that MBP in the lateral ventricle of mice was significantly increased in Catalpol – M - treated EAE mice compared with the PA - treated EAE mice (*P* < 0.01) and increased in Catalpol – M and L - treated EAE mice compared with the Catalpol – H - treated EAE mice (*P* < 0.01, Fig. 7).

**Fig. 7:** The protein expressions of MBP in the brains of mice on Day 18 and Day 40. **a** to **f** show MBP expressions in the cortex of mice on Day40 in NC (*n* = 4), EAE (*n* = 4), EAE+ PA (*n* = 4), EAE + Catalpol–H (*n* = 4), M (*n* = 4) and L (*n* = 4) mice, respectively (scale bar 20 μm). The protein expressions of MBP in the cortex, lateral ventricle and hippocampal DG region of mice were analyzed. Note: ^**^ *P* < 0.01 vs. NC; ^#^ *P* < 0.05, ^##^ *P* < 0.01 vs. EAE; ^◆^ *P* < 0.05, ^◆◆^ *P* < 0.01 vs. EAE+ PA;^▲^ *P* < 0.05, ^▲▲^ *P* < 0.01 vs. EAE + Catalpol–H

A further study was carried out on Day 40. The data showed that the protein expression of MBP in the cortex, and hippocampal DG region of mice was significantly decreased in EAE mice compared with NC mice, respectively (*P* < 0.01). It was significantly increased in PA, Catalpol – H and M - treated EAE mice compared with the EAE mice in the cortex (*P* < 0.05 or *P* < 0.01). The data also showed that MBP was significantly increased in Catalpol – L - treated EAE mice compared with the PA - treated EAE mice in the cortex (*P* < 0.01) and was significantly increased in Catalpol – H, M and L - treated EAE mice compared with the PA - treated EAE mice in the hippocampal DG (*P* < 0.01, Fig. 7).

### Protein expression of Olig1 in the brains of mice on Day 18 and Day 40 PI

Results showed that Olig1 and BrdU separated from each other with IF on Day 18 and Day 40 PI in the cortex. Olig1 was overlapped with cell nucleus (Fig. 8). Compared to NC mice, Olig1 were decreased in the brains on Day 18 and Day 40 PI in EAE mice compared to NC mice (*P* < 0.01). In contrast, Olig1 were significantly increased in PA-treated, Catalpol – H, M and L - treated EAE mice compared to EAE mice in the brains on Day 18 and Day 40 (*P* < 0.05, *P* < 0.01). The protein expression of Olig1 in the cortex of mice was significantly increased in Catalpol-H-treated EAE mice compared with PA-treated EAE mice on Day 18 and Day 40 PI (*P* < 0.01). The protein expression of Olig1 in the cortex of mice was significantly increased in Catalpol – M - treated EAE mice compared with PA-treated, Catalpol – H and L - treated EAE mice on Day 40 (*P* < 0.01, Fig. 8).

**Fig. 8:** Confocal images in the cortex of mice labeled with nucleus (blue) and Olig1 (red). Olig1 was located in nuclear of cells (arrows) and was also present in cytoplasm (arrowheads). A1 to F1 and A2 to F2 show the Olig1+ in the brains of mice on Day 18 and Day 40 in NC (*n* = 4), EAE (*n* = 4), EAE+ PA (*n* = 4), EAE + Catalpol–H (*n* = 4), M (*n* = 4) and L (*n* = 4), respectively (scale bar 100 μm). The protein expressions of Olig1 in the brains of mice were analyzed. Note: ^**^ *P* < 0.01 vs. NC, ^##^ *P* < 0.01 vs. EAE;^◆◆^ *P* < 0.01 vs. EAE+ PA;^▲^ *P* < 0.05, ^▲▲^ *P* < 0.01 vs. EAE + Catalpol–H;^△△^ *P* < 0.01 vs. EAE + Catalpol– M

### Protein expression of Olig2/BrdU in the brains of mice on Day 18 and Day 40 PI

Results showed that Olig2 and BrdU had partial overlap with IF on Day 18 and Day 40 PI. Compared to NC mice, Olig2 were decreased in the brains on Day 18 and Day 40 PI in EAE mice compared to NC mice (*P* < 0.01). In contrast, Olig2 were significantly increased in PA, Catalpol – H, M and L-treated EAE mice compared to EAE mice in the brains on Day 18 and Day 40 (*P* < 0.01). The protein expressions of Olig2 in the hippocampal DG of mice was significantly increased in Catalpol – M - treated EAE mice compared with PA, Catalpol – H and L - treated EAE mice on Day 18 and 40 PI (*P* < 0.01, Fig. 9). Results showed the amplification of Olig2/BrdU with Catalpol – M - treated EAE mice (Fig. 9).

**Fig. 9:** Confocal images in the hippocampus DG of mice double labeled with nucleus (*blue*), Olig2 (*green*) and BrdU (*red*). Olig2 was expressed in cytoplasm of cells (*arrows*). A1 to F1and A2 to F2show the Olig2+/BrdU+ in the brains of mice on Day 18 andDay40 in NC (*n* = 4), EAE (*n* = 4), EAE+ PA (*n* = 4), EAE + Catalpol–H (*n* = 4), M (*n* = 4) and L (*n* = 4) mice, respectively (scale bar 50 μm). The protein expressions of Olig2/BrdU in the brains of mice were analyzed. Note: ^**^ *P* < 0.01 vs. NC, ^##^ *P* < 0.01 vs. EAE; ^◆◆^ *P* < 0.01 vs. EAE+ PA; ^▲^ *P* < 0.05, ^▲▲^ *P* < 0.01 vs. EAE + Catalpol–H, ^△△^ *P* < 0.01 vs. EAE + Catalpol–M

### Protein expression of Olig1/Olig2 in the brains of mice on Day 18 and Day 40 PI

Compared to EAE mice, the protein expressions of Olig1 were increased in the brains on Day 40 PI in Catalpol – M - treated EAE mice (*P* < 0.05). The protein expressions of Olig2 were increased in Catalpol – H, M and L-treated EAE mice compared to EAE mice in the brains on Day 40 (*P* < 0.05). (Figure 10).

**Fig. 10:** A1 to F1 and A2 to F2 show the protein expressions of Olig1/Olig2 in the brains of mice on Day 18 and Day 40 in NC (*n* = 5), EAE (*n* = 5), EAE + PA (*n* = 5), EAE + Catalpol–H (*n* = 5), M (*n* = 5) and L (*n* = 5) mice, respectively. The protein expressions of Olig1/Olig2 in the brains of mice were analyzed. Note: ^#^ *P* < 0.05 vs. EAE; ^◆^ *P* < 0.05 vs. EAE + PA; ^▲^ *P* < 0.05 vs. EAE + Catalpol–H

### Effects of Catalpol on mRNA expression of Olig1 and Olig2 in the brains

The data showed that the mRNA expression of Olig1 in the brains of mice was significantly increased in EAE mice compared with PA-treated EAE mice on Day 18 (*P* < 0.05). The mRNA expression of Olig1 in the brains of mice was significantly increased in Catalpol – H and M - treated EAE mice compared with EAE mice, PA-treated EAE mice and Catalpol – L - treated EAE mice on Day 40 (*P* < 0.01, Fig. 11). Furthermore, the data showed that the mRNA expression of Olig2 in the brains of mice was significantly increased in PA-treated EAE mice compared with EAE mice, Catalpol – H, M and L - treated EAE mice on Day 18. (*P* < 0.01) The mRNA expression of Olig2 in the brains of mice was significantly increased in Catalpol – H and M - treated EAE mice compared with EAE mice, PA and Catalpol – L - treated EAE mice on Day 40. (*P* < 0.01, Fig. 11)

**Fig. 11:** The gene expressions of Olig1 and Olig2 in the brains of mice on Day 18 and 40 in NC (*n* = 5), EAE (*n* = 5), EAE + PA (*n* = 5), EAE + Catalpol–H (*n* = 5), M (*n* = 5) and L (*n* = 5) mice, respectively. Note: ^#^ *P* < 0.05, ^##^ *P* < 0.01 vs. EAE; ^◆◆^ *P* < 0.01 vs. EAE+ PA; ^▲▲^ *P* < 0.01 vs. EAE + Catalpol–H, ^△△^ *P* < 0.01 vs. EAE + Catalpol–M

## Discussion

In this study, EAE was induced by injecting MOG_35–55_ antigen. The features of EAE were confirmed by the observed marked increase in neurological function scores, the existence of inflammatory infiltrates in the brains of EAE mice, and damage to axons and the myelin sheath. We observed the demyelinated fibers were much more tightly bound in EAE mice, which are consistent with previous reports [50, 51]. While treatment with Catalpol permitted the recovery of severity scores and histopathological changes, demyelination even greater recovery following treatment with Catalpol. Catalpol, an iridoid glycoside extracted from Rehmannia, has been shown to be neuroprotective in CNS [35, 37]. These results indicated that Catalpol exerted neuroprotective effects, with the middle dosage of Catalpol having stronger effects than the high and low dosage of Catalpol in the recovery of neurological function scores. Other studies have demonstrated excessive neuroinflammation are detrimental as inhibiting regenerative process including remyelination in vitro and in vivo [52–54]. Concerning Catalpol attenuating inflammatory injury (suppressing microglial and astrocytic activation), Catalpol with an appropriate dosage might enhance remyelination by modulating inflammatory response [55, 56].

To analyze the promoting remyelination mechanisms of Catalpol, we investigated the development of NG2 in the EAE brains. NG2 protein, is essential for remyelination and pericytes, which expressed by OPCs [12]. NG2 play a role in the pathogenesis and progression of MS/EAE [57, 58]. NG2+ cells significantly increased in the brains of the erythropoietin-treated mice compared with that of the EAE mice [59]. The study found that transplantation of human bone marrow stromal cells showed BrdU+ cells expressed NG2+ immunoreactivity, implying that stimulated progenitor and young and mature oligodendrocyte proliferation [60]. The data also showed similar results, Catalpol played a prominent role in increasing NG2 expression of EAE mice, implying that administration of Catalpol enhanced OPCs survival and/or stimulated proliferation of these cells. Meanwhile, the protecting mechanisms of Catalpol on the myelin and axon were related to alleviating the damages in the white and gray matter by the results of MBP in Catalpol treatment groups, especially in the lateral ventricle and hippocampus DG.

We further observed the remyelination mechanisms through which Catalpol affected the mRNA and protein expression of Olig1 and Olig2, in the acute stage and duration stage of EAE. Comparing the EAE mice groups, the neurological function scores decreased in the Catalpol groups which implied that chronic neurological damage could be partly reversed with Catalpol treatments in the duration stage. As the neurological function scores decreased, we also found that gene and protein expressions of Olig1 and Olig2 increased in the Catalpol treatment groups.

Olig1 and Olig2 encode basic helix-loop-helix transcription factors, and were shown to be essential for the remyelination by OPC proliferation and differentiation [61]. Olig1 and Olig2 are two critical transcription factors for both oligodendrocyte development and remyelination [62, 63]. The evidence showed that Olig1 contributed much more to OLs differentiation in the brains, and Olig2 was required for oligodendrogliogenesis in the spinal cord [64–66]. The precursor cells expressing Olig2 had priority to differentiate into OL in the lesion region, and Olig2 was necessary for the specification of OLs postnatally [67, 68]. The Olig2/BrdU double-staining result showed that new formed cells of OPCs and the Olig2 gene were expressed in Catalpol and PA treated groups more than others in nucleus, especially in the surrounding hippocampus and D3V. The reason for this may be that the Olig2 gene is not expressed without lesions in adult mice. This was also not expressed in the normal control group as there was no resulting stimulation. Although it has been proven that the OPCs over-proliferated surrounding lesions in MS patients, the cause of this phenomenon remains unclear, and may be related to the wide use of PA therapy in MS. However, when analyzing the results of Olig1 detection, we confirmed that PA promoted OPCs. These cells proliferated but failed to mature, since Olig1 was poorly expressed in the PA-treatment group. Olig1 can promote the functions of Olig2 [65, 69], and it plays an essential role in the differentiation and remyelination of OLs by maintaining Olig2 expression [67, 70]. Olig1−/− mice were characterized by the normal recruitment of OPCs, but these OPCs failed to differentiate into mature OLs [65]. In the experiment, the data showed that Olig1 was not only expressed in the cytoplasm and nucleus of cells located in the cortex of the brains, but was also expressed in the hippocampus and areas surrounding the lateral ventricle. The high expression in these locations could help naked axons to be myelinating. By analysis of qRT-PCR results, the data showed that Olig1 was expressed at high levels on Day 40.

Th17 cells as a critical pathogenic T cells in pathogenesis of EAE were also counted by FCM [71]. The outcomes indicated the ability of down-regulating Th17 cells with Catalpol treatment performed in EAE course [72]. Considering the modulation of Th17 cells in EAE with Catalpol treatment, one crucial approach of enhancing Olig2 and Olig1 expressions with Catalpol treatment might be down-regulating Th17 cells resultant.

## Conclusion

In summary, the study showed Catalpol could attenuate chronic inflammatory injury and neurological function damage in EAE mice by protecting and regenerating OLs. These positive effects on the OLs might be related to proliferation and differentiation of OPCs by promoting gene and protein expressions of Olig1 and Olig2. This study also indicated one approach of these positive effects responding to the modulation of Th17 which implied that Catalpol had potential as a medication to treat MS.

## Abbreviations

CFA: Complete Freund’ adjuvant
CNS: Central nervous system
DAB: 3,3’-diaminobenzidine tetrahydrochloride
EAE: Experimental autoimmune encephalomyelitis
FCM: Flow cytometric
H&E: Hematoxylin-eosin
IF: Immunofluorescence
IHC: Immunohistochemical
IOD: Integral optical density
MBP: Myelin basic protein
MOG: Myelin oligodendrocyte glycoprotein
MS: Multiple sclerosis
NG: Nerve-glial antigen
OLs: Oligodendrocytes
OPCs: Oligodendrocyte precursor cells
PA: Prednisone acetate
PTX: Pertussis toxin
qRT-PCR: Real-time fluorescent quantitative reverse transcription PCR
SE: Standard error
